# Endoscopic Surgical Treatment of Osteoarthritis and Prognostic Model Construction

**DOI:** 10.1155/2022/1799177

**Published:** 2022-09-05

**Authors:** Qi Su, Guokang Xu

**Affiliations:** Department of Orthopedics, The First People's Hospital of Fuyang District, Hangzhou, China

## Abstract

**Purpose:**

Osteoarthritis (OA) is a degenerative disease of joints. Currently, there is still a lack of effective tools to predict the long-term efficacy of surgical treatment of OA. The purpose of this study was to explore the prognostic factors of endoscopic surgery for OA and to predict the long-term efficacy of this type of surgery for OA by establishing a prognostic model.

**Methods:**

Baseline and follow-up data on 236 OA patients who underwent surgery in our hospital from January 2017 to December 2021 were selected and patients were randomly assigned to a training set (*n* = 165) and a test set (*n* = 71). The Pearson correlation coefficient was used to analyze the correlation between features. Feature selection was performed by recursive feature elimination (RFE) and linear regression. *K*-means clustering analysis was performed on the selected features to obtain the number of output layers. Finally, a single hidden layer error backpropagation (BP)-artificial neural network (ANN) model was established on the training set, and receiver operating characteristic (ROC) curve was drawn on the test set for verification.

**Results:**

Correlation analysis revealed no redundancy among features. RFE and linear regression screened out the features associated with postoperative prognosis under endoscopic surgery: sex, age, BMI, region, morning stiffness time, step count, and osteophyte area. *K*-means clustering yielded that the optimal number of categories was three, the same as the number of categories for the outcome variable. Therefore, a 7-1-3 BP neural network model was established based on these 7 features, and this model could predict the postoperative situation within one year to a relatively accurate extent: area under curve values (AUC) were 0.814, 0.700, and 0.761 in patients with worse, unchanged, and improved conditions one year after surgery, respectively, higher than the multiclass AUC value (0.646).

**Conclusion:**

The prognostic model of endoscopic surgery for OA constructed in this study can well predict the disease progression of patients within one year after surgery.

## 1. Introduction

Osteoarthritis (OA) is a kind of degenerative joint disease that usually occurs in the elderly, and age over 65 years is a clinical risk factor for OA [1]. In addition to age, obesity and joint injury are also common causes of OA [2]. The rising number of years lived with disability (YLD) of OA patients is adding more burdens on the health care and economy in many countries [3]. For OA patients who do not respond to basic treatment or drug therapy, surgery is an alternative to relieve their symptoms [4]. However, according to survey data, only 12.5% of OA patients have effective symptom improvement one to two years after surgery [5]. In-depth study on how to effectively predict the long-term efficacy of surgery for OA patients is still deficient.

Arthroscopic surgery is a routine choice for alleviating OA symptoms and is considered to be effective in improving the clinical symptoms of OA patients [6]. In one study on the effect of arthroscopic repair surgery, Stafford et al. [7] found that the condition of the hip joint of patients undergoing surgical treatment is significantly improved. However, the efficacy of arthroscopic surgery for knee lesions is still controversial. In a placebo-controlled study, the clinical outcome of arthroscopic surgery for knee OA did not significantly improve patients' clinical symptoms compared with drug therapy or placebo [8, 9]. As the efficacy of surgical treatment for OA is affected by many clinicopathological factors, how to select OA patients that are appropriate for surgical intervention needs to be studied.

With the continuous development of machine learning algorithms, artificial neural network (ANN) has been increasingly applied in medical field. Janjic et al. [10] predicted the neural development of premature infants using feed-forward neural networks (fNNs), and their predictive sensitivity on cognitive delay and motor delay in preterm infants reached 85.7% and 76.9%, respectively. Error backpropagation (BP) algorithm-based ANN also plays an important role in the study of immune-mediated diseases [11]. However, few studies have been conducted to predict the long-term outcomes of OA patients undergoing surgical treatment.

Based on the above background, this study intended to analyze the prognostic influencing factors by recursive feature elimination (RFE) and linear regression, based on which we constructed an ANN model to predict the prognosis of hip or knee OA patients after arthroscopic surgery. The purpose of this study was to develop a model that can effectively predict the long-term outcomes of OA patients undergoing surgical treatment and to provide a high-confidence decision-making tool for OA patients' clinical treatment.

## 2. Materials and Methods

### 2.1. Subjects

In this study, 236 OA patients who received surgical treatment in The First People's Hospital of Fuyang District from January 2017 to December 2021 were enrolled. The inclusion criteria were as follows: [1] in line with the clinical manifestations described in the *Guidelines for Diagnosis and Treatment of Osteoarthritis (2018 Edition)* [4]: varying degrees of joint pain and tenderness, joint swelling, limitation of motion, deformity, bone friction, and muscle atrophy; [2] all were diagnosed as knee or hip osteoarthritis by X-ray examination; [3] the patient received endoscopic surgery on the joint for the first time. The exclusion criteria were as follows: [1] coagulation dysfunction; [2] combined with heart, lung, brain, and kidney dysfunction or serious mental illness. The research program was approved by the Medical Ethics Committee of The First People's Hospital of Fuyang District. The informed consent of patients was abandoned since this study was a retrospective study and involved no clear personal information about patients.

### 2.2. Data Collection

Preoperative baseline data of patients were collected. The preoperative baseline data included age, sex, body mass index (BMI), morning stiffness time, Kellgren and Lawrence classification, osteophyte area, step count, site of onset, type of surgery, and the Western Ontario and McMaster Universities Arthritis Index (WOMAC) scores before surgery and one year after surgery. WOMAC is a disease-specific instrument for assessing pain, stiffness, and physical function in patients with hip or knee osteoarthritis [12]. Outcome variables were divided into 3 categories. “Better”: postoperative WOMAC score - preoperative WOMAC score <0; “Maintain”: postoperative WOMAC score - preoperative WOMAC score = 0; “Worse”: postoperative WOMAC score - preoperative WOMAC score >0.

### 2.3. Feature Selection

In the pre-processing stage of data, the correlation between features was calculated first. Then, features with a correlation less than 0.5 were subjected to RFE for secondary screening. RFE is a wrapping feature selection method. Starting from including all features, RFE ranks the importance of all features by establishing a model; the modeling process is repeated after removing the least important features in sequence until the optimal feature subset is screened out [13]. Subsequently, the selected features were used as the input layer to construct the BP-ANN model.

The features selected by RFE were analyzed by *k*-means clustering. The optimal number of classifications obtained by the *k*-means cluster analysis was three categories, which were the same as the outcome variables set in this study. Therefore, the output layer was 3 in the establishment of the BP neural network.

### 2.4. Machine Learning Model Construction and Solving Algorithms

To predict the long-term efficacy of endoscopic surgery for OA, a feed-forward neural network was used for modeling. The patients were randomly assigned to a training set (*n* = 165) and a test set (*n* = 71), and a single hidden layer BP-ANN model was established with the training set.

In order to predict the long-term efficacy of endoscopic surgery for OA, we adopted fNN for modeling. fNN is a one-way multi-layer neural network, whose structure includes input layer, hidden layer, and output layer (Figure 1). Parameters of the model mainly include weights of connections between layers and thresholds of both hidden layer and output layer (*ω*, *v*, *θ*, and *γ* in Figure 1). In this study, the features obtained from RFE were brought into the neurons in the input layer and solved by BP algorithm. During training, we set the learning rate to 0.001 and the BP algorithm adjusts parameters of models based on the idea of gradient descent method until the accuracy of the result reaches the required level [14].

### 2.5. Model Verification

The receiver operating characteristic (ROC) curve was used to evaluate the established model in the test set. Since the purpose of the model was to predict a result of three-way classification, we plotted the ROC curve of each category and the overall ROC curve to reflect the accuracy of prediction with the area under curve (AUC).

### 2.6. Statistical Analysis

The selection of features in this study was performed using “caret” package, and the establishment and solving of the neural network model depended on the “nnet” package in R package. In the modeling process, the number of neurons in the hidden layer was set in turn from small to large. After ten-fold cross verification, the number of neurons corresponding to the minimum mean squared error (MSE) was taken. ROC curve plotting was completed with the “pROC” package. Continuous variables conforming to normal distribution were represented as mean ± standard deviation, while continuous variables not conforming to normal distribution were represented with median value (interquartile range). Counting variables were represented as *n*, %.

## 3. Results

### 3.1. Patient Features

A total of 236 patients were included in the study, with an age of 67.00 (60.00, 70.00) years, 38.1% male and 61.9% female, median BMI of 24.51 (21.26, 26.60). The number of patients with morning stiffness time less than or equal to 10 min, within 10-20 min, and more than 20 min was 142, 43, and 51, respectively. Other articular-related information, including Kellgren and Lawrence classification, osteophyte area, mean daily step count, lesion status, and surgical type, are shown in Table 1.

### 3.2. Feature Selection

To test the redundancy between features, we calculated the Pearson correlation coefficient between features and obtained the correlation matrix (Table 2). The absolute values of the correlation coefficients between patient features were all <0.5, so there was no redundancy between features.

Linear regression was used to calculate the importance of features, and the results showed that the importance of sex, age, BMI, and other features decreased in descending order (Figure 2(a)). The results of RFE screening showed that the root mean square error (RMSE) of the model reached the minimum value when seven features were retained (Figure 2(b)). These features included sex, age, BMI, region, morning stiffness time, step count, and osteophyte area, and the minimum RMSE was 0.687. Therefore, these 7 features were used as the input layer for building the BP-ANN model.

Furthermore, the factors screened by RFE method were subjected to cluster analysis. The optimal number of clusters of *k*-means was determined by the total cluster sum of squares. The optimal results were obtained when the number of clusters was 3 (Figures 3(a) and 3(b)), which was the same as the cluster number of outcome variables in this study.

### 3.3. BP-ANN Model

Seven features (sex, age, BMI, region, morning stiffness time, step count, and osteophyte area) screened out by the RFE method in the training set were used as the input layer, and three types of outcome variables as the output layer to build a single hidden layer neural network model. When the maximum number of iterations was set to 200, a neural network model was established by BP algorithm (Figure 4). The maximum number of iterations was not achieved when the computation stopped.

### 3.4. Model Evaluation

After the BP neural network was trained on training set, the predicted classification of the test set was obtained, and then the accuracy of the model was verified with the test set and the ROC curve of the model validation results in the training set was drawn (Figure 5). The ROC curve illustrated that the AUC values of the model in patients with OA worse (0.814), maintain (0.700), and better (0.761) were higher than the multiclass AUC value (0.646), indicating high accuracy of the model and its potential for prediction of one-year postoperative outcome in patients with OA.

## 4. Discussion

In this study, patients with hip or knee OA after arthroscopic surgery were analyzed, and the prognostic influencing factors were screened by RFE. The RMSE value of the linear model reached the minimum value of 0.687 when 7 features were selected, and these 7 clinical features included sex, age, BMI, region, morning stiffness time, average step count, and osteophyte area. Subsequently, a 7-1-3 type BP-ANN model was established by using these 7 influencing factors as input variables to predict the prognosis one year after surgery.

Seven characteristics including sex, age, BMI, region, morning stiffness time, step count, and osteophyte area were found to have an impact on the prognosis of surgery through linear regression and RFE method, and their importance decreased in order. Abramoff et al. [15] reported that the incidence of OA increases with age and is the greatest risk factor for OA. Additionally, BMI (overweight/obesity) is also associated with the progression of hip/knee OA in clinical practice [16–18]. Most studies indicated that women are more likely to develop OA than men [19–21]. Other risk factors for OA are race, morning stiffness, osteophytes, and limited motion [15, 22–24]. In this study, region, morning stiffness time, step count, and osteophyte area ranked relatively low, and their influence on OA needs further analysis. Knee joint and hip joint are commonly involved joints in OA [2]. Patients with this type of OA often have difficulties in walking when the condition is serious, which greatly reduced their quality of life [2]. As the number of involved joints increases, the walking ability of patients becomes worse [2]. Through one-way ANOVA or *t*-test, Kwon et al. [25] selected knee OA patients' clinical features for constructing an artificial intelligence network model. This is different from the strategy of our study. During feature selection, the importance of each feature was first calculated by the linear regression model, and then the RFE algorithm was used to remove the least important features to obtain 7 clinical features, which were selected as the input layer to build the BP-ANN model. When 7 clinical features were screened out, the RMSE value reached the minimum. A related study believes that arthroscopic hip surgery is relatively safe because of its low incidence of postoperative complications [26], while the benefits of arthroscopic knee surgery remain controversial [27]. Unfortunately, we did not compare the hazard ratio of hip and knee surgeries in the present study, and therefore, we cannot discuss the clinical benefits of either procedure.

In the present study, BP-ANN network was used to predict the disease progression of OA patients one year after surgery. Firstly, the correlation matrix analysis was carried out on the clinical characteristics of patients by the Pearson correlation coefficient, and the results presented no redundancy among characteristics. Then, combined with linear regression and RFE to screen their importance, 7 feature factors related to prognosis were obtained. *K*-means clustering revealed the number of classifications was 3. Subsequently, a “7-1-3” BP-ANN model was constructed based on these 7 features on the training set. Finally, the ROC curve verified high prediction accuracy of the model. Halilaj et al. [28] also carried out research related to the progress of OA using ANN model. Their study conducted cluster analysis on the clinical features of OA patients, and based on the clustering results, a Least Absolute Shrinkage and Selection (LASSO) model was developed to predict changes in joint spaces and WOMAC scores, with predictive AUC of 0.86 and 0.95, respectively. This is similar to the results of our study. Our findings may generate new insights into the construction of prognostic models for OA patients. In addition, by using machine learning algorithm, Sniderman et al. [29] predicted the outcomes (including hip disability and osteoarthritis outcome score (HOOS) 3 months after surgery) of patients undergoing hip replacement. Their study constructed a model for prediction by LASSO algorithm. Different from their study, our study integrated patients with OA of hip joint and knee joint and included three surgical methods: articular cartilage repair, arthroscopic debridement, and osteotomy. Based on the analysis results of our study, surgical method was not a significant clinical feature that affected the prognosis of OA patients. Currently, various researchers are attempting to apply artificial intelligence algorithms to multiple OA-related fields, such as the screening of OA clinical pathologic factors, prediction of postoperative efficacy, and OA pathological classification. However, developing more efficient and accurate algorithms and models that can guide clinicians to make better decisions is still needed.

To conclude, this study found that sex, age, BMI, region, morning stiffness time, step count, and osteophyte area were prognostic influencing factors for arthroscopic surgery and established a neural network structured prognostic model. However, due to insufficient follow-up data, we only conducted a one-year postoperative study, and the features included in the study were limited. In the future, the follow-up data at multiple time points can be used to establish a model to predict the outcome of surgery at different times. In addition, the inclusion of more factors will improve the screening of prognostic factors. The achievements of these improvements will provide more favorable evidence for the treatment of OA.

## Figures and Tables

**Figure 1:** Structure of fNN. Note: **x**_1_, ⋯, **x**_**n**_ ,**b**_1_, ⋯, **b**_**k**_, and **y**_1_, ⋯, **y**_**m**_ are neurons of input layer, hidden layer, and output layer, respectively; **ω**_11_, ⋯, **ω**_**nk**_ and **v**_11_, ⋯, **v**_**km**_ are the connection weights between input layer and hidden layer and between hidden layer and output layer; **θ**_1_, ⋯, **θ**_**k**_ and **γ**_1_, ⋯, **γ**_**m**_ are the thresholds of the hidden layer and the output layer, respectively.

**Figure 2:** Feature selection by linear regression. (a) Order of importance of all features in linear regression; (b) Selection of optimal number of retained features by RFE. Note: RMSE: root mean square error.

**Figure 3:** *K*-means clustering. (a) Total cluster sum of squares at different number of clusters (*k*). (b) Clustering results when the number of clusters *k* = 3. Note: PC: primary component.

**Figure 4:** Neural network model.

**Figure 5:** ROC curves of model clustering results. Note: FTR: false positive rate; TPR: true positive rate.

**Table 1:** Baseline data and pathological features of patients.

Feature	Description
Sample size, *n*	236
Age, years	67.00 (60.00, 70.00)
*Sex, %*	
Female	146 (61.9)
Male	90 (38.1)
BMI	24.51 (21.26, 26.60)
*Morning stiffness time, %*	
≤10 minutes	142 (60.2)
> 10 minutes and ≤ 20 minutes	43 (18.2)
>20 minutes	51 (21.6)
*Kellgren and Lawrence classification, %*	
I	18 (7.6)
II	84 (35.6)
III	83 (35.2)
IV	51 (21.6)
Osteophyte area, *mm*^2^	5.483 (4.030, 6.830)
*Daily average step count, %*	
≤3000	57 (24.2)
>3000 and ≤8000	101 (42.8)
>8000	78 (33.1)
*Involved parts, %*	
Hip joint	128 (54.2)
Knee joint	108 (45.8)
*Number of joints involved, %*	
Unilateral	132 (55.9)
Bilateral	104 (44.1)
*Surgical type, %*	
Articular cartilage repair	84 (35.6)
Arthroscopic debridement	117 (49.6)
Osteotomy	35 (14.8)

**Table 2:** Correlation matrix between features.

	Age	Sex	BMI	Morning stiffness time	Region	KL score	Osteophyte area	Step count	Joint	Involved joint	Surgical type	Evaluation
Age	1.000	-0.062	0.008	-0.106	-0.010	0.003	0.021	-0.048	0.021	0.044	0.068	-0.293
Sex	-0.062	1.000	-0.036	0.029	0.152	-0.056	-0.083	0.023	-0.056	0.006	0.073	0.319
BMI	0.008	-0.036	1.000	0.022	0.087	0.007	-0.010	-0.182	0.002	0.122	0.089	-0.235
Morning stiffness time	-0.106	0.029	0.022	1.000	-0.012	0.031	0.009	-0.027	0.069	0.011	0.062	0.120
Region	-0.010	0.152	0.087	-0.012	1.000	-0.043	0.025	0.225	0.147	-0.179	-0.063	0.172
KL score	0.003	-0.056	0.007	0.031	-0.043	1.000	0.059	0.033	-0.081	-0.073	-0.262	-0.040
Osteophyte area	0.021	-0.083	-0.010	0.009	0.025	0.059	1.000	0.080	-0.074	-0.025	-0.039	-0.051
Step count	-0.048	0.023	-0.182	-0.027	0.225	0.033	0.080	1.000	0.072	0.054	-0.105	0.152
Joint	0.021	-0.056	0.002	0.069	0.147	-0.081	-0.074	0.072	1.000	0.041	0.005	0.024
Involved joint	0.044	0.006	0.122	0.011	-0.179	-0.073	-0.025	0.054	0.041	1.000	0.083	-0.060
Surgical type	0.068	0.073	0.089	0.062	-0.063	-0.262	-0.039	-0.105	0.005	0.083	1.000	-0.016
Evaluation	-0.293	0.319	-0.235	0.120	0.172	-0.040	-0.051	0.152	0.024	-0.060	-0.016	1.000

Note: BMI: body mass index; KL score: Kellgren-Lawrence classification.

## Data Availability

The data that support the findings of this study are available on request from the corresponding author. The data are not publicly available due to privacy or ethical restrictions.
